# Combination of sorafenib and gadolinium chloride (GdCl3) attenuates dimethylnitrosamine(DMN)-induced liver fibrosis in rats

This article has been retracted.

**DOI:** 10.1186/s12876-015-0380-5

**Published:** 2015-11-16

**Authors:** Cheng Liu, Zongguo Yang, Lei Wang, Yunfei Lu, Bozong Tang, Hui Miao, Qingnian Xu, Xiaorong Chen

**Affiliations:** 1 Department of Traditional Chinese Medicine, Shanghai Public Health Clinical Center, Shanghai, 201508 China; 2 Laboratory of Molecular Pathology, Central Laboratory, Putuo Hospital, Shanghai University of Traditional Chinese Medicine, Shanghai, 200062 China; 3 Department of Hepatology, Affiliated hospital of Shandong University of Trasitional Chinese Medicine, 250014 Jinan, China

**Keywords:** Hepatic stellate cells, Sinusoidal endothelial cells, Kupffer cells, Liver fibrosis

## Abstract

**Background/aims:**

Liver sinusoidal endothelial cells (SECs), hepatic stellate cells (HSCs) and Kupffer cells (KCs) are involved in the development of liver fibrosis and represent a potential therapeutic target. The therapeutic effects on liver fibrosis of sorafenib, a multiple tyrosine kinase inhibitor, and gadolinium chloride (GdCl3), which depletes KCs, were evaluated in rats.

**Methods:**

Liver fibrosis was induced in rats with dimethylnitrosamine, and the effects of sorafenib and/or GdCl3 in these rats were monitored. Interactions among ECs, HSCs and KCs were assessed by laser confocal microscopy.

**Results:**

The combination of sorafenib and GdCl3, but not each agent alone, attenuated liver fibrosis and significantly reduced liver function and hydroxyproline (Hyp). Sorafenib significantly inhibited the expression of angiogenesis-associated cell markers and cytokines, including CD31, von Willebrand factor (vWF), and vascular endothelial growth factor, whereas GdCl3 suppressed macrophage-related cell markers and cytokines, including CD68, tumor necrosis factor-α, interleukin-1β, and CCL2. Laser confocal microscopy showed that sorafenib inhibited vWF expression and GdCl3 reduced CD68 staining. Sorafenib plus GdCl3 suppressed the interactions of HSCs, ECs and KCs.

**Conclusion:**

Sorafenib plus GdCl3 can suppress collagen accumulation, suggesting that this combination may be a potential therapeutic strategy in the treatment of liver fibrosis.

**Electronic supplementary material:**

The online version of this article (doi:10.1186/s12876-015-0380-5) contains supplementary material, which is available to authorized users.

## Background

Liver fibrosis, as the final common endstage of most chronic liver diseases, is triggered by chronic liver injury caused by various etiologies including viral infection, cholestasis, metabolic diseases and alcohol abuse [1, 2]. Chronic liver injury and the ensuing inflammatory responses result in the activation of quiescent HSCs, which proliferate and undergo phenotypical and morphological changes, subsequently turning into characteristic myofibroblasts with up-regulated alpha-smooth muscle actin (α-SMA) expression and ECM production [3–6]. Although the mechanisms underlying the progression of hepatic fibrosis are fairly well understood, safe and effective antifibrotic therapies are needed for patients with chronic liver diseases [7].

Sorafenib is a multiple receptor tyrosine kinase inhibitor targeting the Raf/ERK signaling pathways, as well as receptor tyrosine kinases such as vascular endothelial growth factor receptor (VEGFR) and platelet-derived growth factor receptor (PDGFR)-β [8]. Sorafenib induces apoptosis in various tumor cell lines and used to treat patients with advanced hepatocellular carcinoma (HCC), cholangiocellular carcinoma and portal pressure [9, 10]. Sorafenib was recently reported to suppress collagen accumulation in rats with liver fibrosis and portal hypertension [11, 12]. Another study reported, however, that sorafenib can induce liver damage, while reducing the number of activated HSCs and intrahepatic vascular resistance in cirrhotic livers [13].

Macrophages play a key role in inflammation associated with liver fibrosis. The *in vivo* role of macrophages has been assessed by depleting macrophage populations with the macrophage apoptosis inducers gadolinium chloride (GdCl3) and liposome-encapsulated dichloromethylene bisphosphonate (Cl2MBP). GdCl3 has been found to reverse dimethylnitrosamine (DMN)-induced rat liver fibrosis while increasing the expression of matrix metalloproteinases (MMPs) by KCs [14, 15]. However, we found that GdCl3 did not reduce liver fibrosis significantly because of its proinflammatory effects on lung macrophages [16]. Taken together, these findings indicate that liver fibrosis is a systematic disease associated with specific microenvironments, including interactions among HSCs, ECs and KCs. This study analyzed the effects of sorafenib plus GdCl3 on DMN-induced liver fibrosis in rats.

## Methods

### Materials and chemicals

Sorafenib (Alexis Biochemicals, San Diego, CA, USA) was dissolved in 1:1:6 mixture composed of Cremophor EL (Sigma-Aldrich, St. Louis, MO, USA), ethanol and water. GdCl3 was from Sigma-Aldrich (Catalog No. 203289) and DMN was from Wako (Osaka, Japan; Catalog No. 149–05882). Sirius red was obtained from Polysciences (Sigma-Aldrich; Catalog No. 365548) and dissolved in saturated picric acid (Chroma, Munster, Germany). SYBR Green Supermix was from Thermo Fermentas (Glen Burnie, MD, USA), and prestained protein marker was purchased from New England Biolabs (Beijing, China). All primary antibodies were from Santa Cruz (Santa Cruz, CA, USA).

### Ethics statement

All of the study protocols complied with the current ethical considerations of Shanghai Public Health Clinical Center’s Animal Ethic Committee and the procedural and ethical guidelines of the Chinese Animal Protection Act, which is in accordance with the National Research Council criteria. All animal experiments and procedures were reviewed and approved by the Institutional Animal Care and Use Committee (IACUC) of Shanghai Public Health Clinical Center and were performed in accordance with the relevant guidelines and regulations.

### Animal experiments

Wistar rats weighing 160–180 g were provided by the Central Animal Care Facility of Shanghai Public Health Clinical Center (Permission No: SCXK 2007–0006). All animals were cared for humanely, in compliance with the Chinese Animal Protection Act and National Research Council criteria.

Rats were randomized into two groups, with 40 animals intraperitoneally injected with DMN (10 mg/kg body weight) for three consecutive days per week for 4 weeks [17, 18], and ten control rats were injected with equal volumes of physiological saline. At the beginning of the third week, the DMN-treated rats were further randomized into four groups, with ten each receiving sorafenib (1 mg/kg/day by gavage); GdCl3, at a dose of 7 mg/kg in isotonic saline [14] twice weekly for 2 weeks, administered through the tail vein; sorafenib plus GdCl3; or vehicle, as well as being continued on DMN for another 2 weeks, as above. The dose of GdCl3 was set at 7 mg/kg, because this dose had no effect on liver enzyme activity but was reported to inhibit Kupffer cell phagocytosis [19]. At the end of the fourth week, all the rats were sacrificed under 2 % sodium pentobarbital anesthesia, and all efforts were made to minimize suffering. Some of these samples were directly transferred to buffered 10 % formaldehyde solution for paraffin embedding, whereas the remainder were frozen in liquid nitrogen and stored for later analyses.

### Serum biochemistry

Serum was prepared by centrifugation at 3000 rpm at 4 °C and stored at −80 °C. Serum concentrations of alanine aminotransferase (ALT), aspartate aminotransferase (AST), albumin (ALB) and total bilirubin were measured by the Clinical Laboratory of Shanghai Public Clinical Health Center.

### Hydroxyproline determination

Hepatic hydroxyproline (Hyp) content was used as an indirect measure of tissue collagen content. Hepatic hydroxyproline content was measured using a hydroxyproline detection kit (Jiancheng Institute of Biotechnology, Nanjing, China) according to the manufacturer’s instructions. Hydroxyproline content was expressed as μg/gram of liver wet weight.

### Liver histology

Liver tissues from the right lobe of the liver of each rat were fixed in 4 % buffered paraformaldehyde, and dehydrated in a graded alcohol series. Following the xylene treatment, the specimens were embedded in paraffin blocks, cut into 5 μm-thick sections and placed on glass slides. The sections were stained with HE and Sirius red. The area of Sirius red-positive staining was quantified using a computer-aided image analysis software image-pro plus version 6.1 (MediaCybernetics, USA).

### Immunohistochemistry

After deparaffinization and dehydration, microwave antigen retrieval was performed for 5 min, followed by peroxidase quenching with 0.6 % H_2_O_2_ in phosphate-buffered saline (PBS) for 15 min. The sections were subsequently blocked with 5 % bovine serum albumin (BSA) for 30 min and incubated overnight at 4 °C with 1:100 dilutions of primary antibodies to vWF, CD68, and α-SMA. Negative control sections were treated identically, except for omission of the primary antibodies. After washing in PBS, the sections were incubated with biotinylated secondary antibodies for 30 min.

### Protein extraction and western blot analysis

Protein was extracted and western blot analysis was performed as described [18]. Briefly, aliquots of tissue lysates containing 50 μg protein were electrophoresed on 10–12 % sodium dodecyl sulfate-polyacrylamide gels and transferred to nitrocellulose membranes. The membranes were blocked with 5 % BSA and incubated with 1:100 dilutions of antibodies overnight at 4 °C, followed by incubation with horseradish peroxidase-conjugated goat anti-mouse antibody (1:5000) and visualization by enhanced chemiluminescence (Pierce, Rockford, IL, USA) using Kodak films (Kodak, Rochester, NY, USA).

### Quantitative real-time PCR

RNA isolation, reverse transcription, and RT-PCR were performed as previously described [20]. Briefly, total RNA was isolated from 50 mg flash-frozen liver tissue using RNeasy-easy kit (Qiagen, Hilden, Germany, Cat: 74104), followed by reverse transcription of 1 μg aliquots of RNA (Fermentas). Quantitative polymerase chain reaction (PCR) was performed on an ABI7700 Sequence detector (Applied Biosystems, Rotkreuz, Switzerland using the primer sequences shown in Additional file 1: Table S1. The expression of each gene was normalized relative to that of 18S rRNA using the delta–delta cycle threshold method.

### Laser confocal microscopy

Liver samples were assessed grossly, immersed immediately in Tissue-Tek OCT, snap-frozen in liquid nitrogen; and cut into 5 μm. The cryosections were stained sequentially with different combinations of antibodies, resulting in tricolor labeling. Imaging results were analyzed using a Leica (Mannheim, Germany) DMIRBE inverted stand and a Leica TCS2MP confocal system.

### Statistical analysis

Each experiment was performed at least three times independently. Results are expressed as mean ± S.D. All statistical analyses were performed using SPSS software version 18.0. Differences between two groups were compared with a two-tailed unpaired *t* test. Differences between multiple groups were compared by one-way analysis of variance with post hoc Tukey tests, with *p* < 0.05 considered statistically significant.

## Results

### Effects of sorafenib plus GdCl3 on liver function

During drug intervention, two rats died in the 4 week DMN group, and one in the GdCl3 group. Animal body, liver, spleen weights were monitored during the formation of liver fibrosis (Additional file 1: Table S2). Compared with control rats, body, and liver weights decreased significantly in the 4 week DMN group (*p* < 0.01), whereas the spleen weight in the 4 week DMN rats increased significantly (*p* < 0.01). the combination of sorafenib with GdCl3 significantly increase liver weight (*p* < 0.05) and decrease spleen weight (*p* < 0.01) compared with 4 week DMN rats.

Rats treated for 4 weeks with DMN developed hepatic injury, as evidenced by significantly higher plasma concentrations of AST, ALT, and total bilirubin (TBil) and a significantly lower concentration of ALB compared with normal control rats (*p* < 0.01 each). While treatment with either sorafenib or GdCl3 had no effect on these plasma protein concentrations (Additional file 1: Table S3), the combination of sorafenib with GdCl3 significantly ameliorated the increases in ALT, AST, and TBil, and the decrease in ALB (*p* < 0.05 or *p* < 0.01) indicating there were synergistic action when combination sorafenib with GdCl3.

### Effects on hepatic histopathological changes

In the liver, there was normal lobular architecture, with the central vein and radiating hepatic cords in the livers of control rat (Fig. 1a). In the 4 week DMN group, the liver sections revealed collagen fiber deposition, marked cirrhosis, and severe centrilobular necrosis. We observed marked reduction in the thickening of the collagen bundles in the combination treatment (S + G) group.

**Fig. 1:** Effects of sorafenib and/or GdCl3 on histological changes of rat livers. **a** Histological images of rat livers stained with HE (magnification X200). **b** Histological images of rat livers stained with Sirius red (magnification X100). **c** qualification of Fig. 1b. **d** Liver Hyp content. The number in HE, Sirius red staining, and Hyp detection was as the same as the animal number in each group. All results are expressed as mean ± S.D. *, *p* < 0.05; ** *p* < 0.01 vs 4 W. Control, vehicle alone; 4 W, DMN for 4 weeks; S, DMN for 4 weeks plus sorafenib for 2 weeks; G, DMN for 4 weeks plus GdCl3 for 2 weeks; S + G, DMN for 4 weeks plus sorafenib and GdCl3 for 2 weeks

Liver fibrosis was quantitatively assessed by morphometric examination of liver sections incubated with 0.1 % Sirius red, which specifically stains collagen. Little collagen was present in normal liver, except around the small central venous walls (Fig. 1b). In contrast, the livers of rats treated for 4 weeks with DMN showed marked distortion of architecture, including portal and lobular bridging fibrosis, cirrhotic nodule formation, and thickened reticulum fibers joining the central areas. Treatment of DMN-treated rats with sorafenib plus GdCl3 significantly decreased liver fibrosis (Fig. 1b and c).

Changes in Hyp content in the liver are considered an index of collagen metabolism and provide valuable information about the biochemistry and pathology of liver fibrosis. Rats treated with DMN showed a significant, 3.2-fold increase in Hyp content, expressed as μg/g of liver tissue (*p* < 0.01), compared with control rats (Fig. 1d), a finding consistent with the marked cirrhosis and accumulation of collagen bundles in the liver observed on histopathological examination. Treatment of rats with sorafenib or GdCl3 slightly reduced the Hyp content in liver (*p* > 0.05), whereas treatment with both resulted in a significant decrease (*p* < 0.05) in liver Hyp, suggesting that combination therapy ameliorated hepatic collagen deposition in DMN-induced liver injury.

### Effect of sorafenib plus GdCl3 on hepatic angiogenesis-related factors

Aberrant angiogenesis has been implicated in the progression of hepatic fibrosis and is considered a major determinant of hepatic dysfunction and irreversibility in cirrhosis [21]. Incubation of tissue sections with antibody to vWF showed very weak staining in control rats, whereas rats treated with DMN for 4 weeks showed an irregular vascular pattern in the portal/periportal areas of the expanding portal tracts. Treatment with sorafenib alone inhibited vessel formation in portal and periportal areas, whereas GdCl3 alone did not markedly inhibit vWF expression. The combination of sorafenib plus GdCl3 significantly reduced vWF expression, indicating that this inhibitory effect was due to sorafenib. Real-time RT-PCR showed that treatment with DMN for 4 weeks increased CD31 mRNA expression about 7-fold compared with control rats. Sorafenib treatment of DMN-treated rats significantly reduced CD31 mRNA expression compared with rats treated with DMN (*p* < 0.01), whereas GdCl3 had little effect on CD31 mRNA expression (Fig. 2b). Sorafenib plus GdCl3 significantly reduced CD31 mRNA expression.

**Fig. 2:** Effect of sorafenib and/or GdCl3 blockage on angiogenesis in DMN-induced liver fibrosis *in vivo*. **a** vWF immunohistochemistry (magnification X400, *n* = 4). **b** Levels of mRNAs encoded by genes related to angiogenesis (*n* = 6). **c** the Expression of CD31, VEGF, Ang1, VCAM1 was analyzed using western blot (*n* = 6). Control, vehicle alone; 4 W, DMN for 4 weeks; S, DMN for 4 weeks plus sorafenib for 2 weeks; G, DMN for 4 weeks plus GdCl3 for 2 weeks; S + G, DMN for 4 weeks plus sorafenib and GdCl3 for 2 weeks. The negative control consisted of samples from DMN-treated animals in the absence of primary antibody. All results reported as mean ± S.D. *p < 0.05; **p < 0.01 vs 4 W

Treatment with DMN significantly enhanced the expression of VEGF, Ang1 and VCAM1 mRNAs compared with control rats, with sorafenib treatment ameliorating these effects and GdCl3 having a slight effect. Sorafenib plus GdCl3 reduced the expression of VEGF, Ang1 and VCAM1 mRNAs significantly compared with DMN-treated rats.

Western blotting with antibodies to CD31, VEGF, Ang 1 and VCAM yielded similar results (Fig. 2c). Taken together, these results showed that liver SECs were important for DMN-induced liver fibrosis. The effects of sorafenib plus GdCl3 on angiogenesis and related factors were likely due to sorafenib, with GdCl3 having little effect.

### Sorafenib plus GdCl3 inhibits proinflammatory cytokines

KCs synthesize a variety of mediators, such as proinflammatory cytokines, chemokines, leukotrienes and reactive oxygen species (ROS), fulfilling a crucial role in immune responses in the liver [22]. KCs inhibition has been shown to protect against hepatic injury, including ischemia/reperfusion injury, alcohol-induced injury, and injuries induced by certain toxicants, such as cycloheximide [23]. While low levels of CD68-positive KCs were present in hepatic sinusoids of control livers, DMN treatment for 4 weeks enhanced the numbers of KCs strongly positive for CD68 in hepatic sinusoids, as well as in portal areas and areas adjacent to fibrotic septa (Fig. 3a). Although sorafenib treatment did not reduce CD68 expression, GdCl3 inhibited CD68 expression significantly. Similarly, real-time RT-PCR showed that DMN treatment upregulated CD68 mRNA expression about 8.8-fold (Fig. 3b); again, although sorafenib had little effect on CD68 mRNA level, GdCl3 reduced CD68 mRNA expression significantly, as did the combination of sorafenib plus GdCl3. Western blotting for CD68 protein yielded similar results (Fig. 3c).

**Fig. 3:** Effects of sorafenib and/or GdCl3 blockage on *in vivo* expression of proinflammatory cytokines in liver fibrosis. **a** CD68 immunohistochemistry (magnification X 400, *n* = 4). **b** Levels of mRNA encoded by genes encoding proinflammatory cytokines in rats with DMN-induced fibrosis (*n* = 6). **c** The Expression of CD68, TNF-α, IL1β, CCL2 was analyzed using western blot (*n* = 6). Control, vehicle alone; 4 W, DMN for 4 weeks; S, DMN for 4 weeks plus sorafenib for 2 weeks; G, DMN for 4 weeks plus GdCl3 for 2 weeks; S + G, DMN for 4 weeks plus sorafenib and GdCl3 for 2 weeks. Results reported as mean ± S.D. *p < 0.05; **p < 0.01 vs 4 W

TNF-α, IL-1β and CCL2 are mainly derived from KCs after liver injury. Real-time RT-PCR showed that 4 weeks of treatment with DMN increased TNF-α mRNA expression about 40-fold (*p* < 0.01) (Fig. 3b). Although sorafenib alone had little effect on TNF-α mRNA level, the combination of sorafenib plus GdCl3 markedly reduced TNF-α mRNA. These findings were further confirmed by western blotting (Fig. 3c).

Taken together, these results showed that KCs were activated during DMN-induced liver fibrosis. Although sorafenib alone could not significantly inhibit KC activation or the production of proinflammatory cytokines, the combination of sorafenib plus GdCl3 suppressed these proinflammatory responses.

### Effect of sorafenib plus GdCl3 on hepatic pro-fibrotic factor expression

Sustained deposition of extracellular matrix mainly results from the activation of HSCs. We therefore assessed the correlation between collagen accumulation and HSC activation by analyzing the expression of α-SMA, a marker of activated HSCs, in liver sections. Although only vascular smooth muscle cells were positive for α-SMA in control rats, the number of α-SMA-positive HSCs was markedly increased after 4 weeks of treatment with DMN (Fig. 4a). Either sorafenib or GdCl3 alone decreased α-SMA expression, findings confirmed by real-time RT-PCR and western blotting (Fig. 4b).

**Fig. 4:** Effects of sorafenib and/or GdCl3 on *in vivo* expression of pro-fibrotic factors in rat liver fibrosis. **a** α-SMA immunohistochemistry (magnification X 200, *n* = 4). **b** Levels of mRNA encoded by genes encoding factors associated with fibrosis sis (*n* = 6). **c** the Expression of α-SMA, TIMP1, TGF-β1, COL1 was analyzed using western blot (*n* = 6). Control, vehicle alone; 4 W, DMN for 4 weeks; S, DMN for 4 weeks plus sorafenib for 2 weeks; G, DMN for 4 weeks plus GdCl3 for 2 weeks; S + G, DMN for 4 weeks plus sorafenib and GdCl3 for 2 weeks. Results reported as mean ± S.D. * *p* < 0.05; ** *p* < 0.01 vs 4 W

The expression levels of TGF-β1, TIMP-1 and Col1 (α1) were markedly higher in DMN-treated than in control rats. The sorafenib or GdCl3 alone could inhibit these profibrotic factor to some extent (there were no significant) the combination of sorafenib plus GdCl3 markedly reduced their expression.

Taken together, these results confirm that DMN activates HSCs and induces the accumulation of extracellular matrix, which may facilitate or result in liver fibrosis. The combination of sorafenib plus GdCl3 significantly inhibited HSC activation and reduced liver fibrosis development.

### Effects of sorafenib plus GdCl3 on interactions of HSC, KC, and SEC

The pathophysiological involvement of HSCs, KCs, and LSECs in DMN-induced liver fibrosis was investigated by immunochemically assessing the co-localization of α-SMA, CD68, and vWF by confocal microscopy. Tricolor immunofluorescence staining of liver sections from rats treated for 4 weeks with DMN showed CD68^+^ KCs near or directly adhering to α-SMA^+^ HSCs in the sinusoids and portal areas (Fig. 5). Sorafenib markedly reduced vWF expression, whereas GdCl3 reduced CD68 expression and the interactions of HSCs and KCs. These results collectively demonstrated that sorafenib combined with GdCl3 inhibited interactions among HSCs, SECs and KCs, cells that play key roles in liver fibrosis.

**Fig. 5:** Effects of sorafenib and/or GdCl3 on interactions of HSCs, KCs and SECs in DMN-induced liver fibrosis in rats. Hepatic cryosections were stained with antibodies against α-SMA (blue), CD68 (*red*), and vWF (*green*) (magnification X400, *n* = 3). 4 W, DMN for 4 weeks; S, DMN for 4 weeks plus sorafenib for 2 weeks; G, DMN for 4 weeks plus GdCl3 for 2 weeks; S + G, DMN for 4 weeks plus sorafenib and GdCl3 for 2 weeks

## Discussion

Angiogenesis and inflammation play important roles in the development of liver fibrosis, making them potential therapeutic targets. Since the anti-fibrotic effects of sorafenib and GdCl3 in the progression of liver fibrosis are unclear, we assessed the *in vivo* therapeutic effects of this combination in DMN-induced liver fibrosis. We found that sorafenib plus GdCl3 achieved effects superior to those of either agent alone, improving liver function and reducing hydroxyproline content. Furthermore, this combination treatment was simultaneously directed against several targets, including angiogenic and proinflammatory factors.

Advanced fibrosis and cirrhosis represent the main pathophysiological consequences of chronic liver disease and can lead to life-threatening clinical sequelae [24]. The major mechanisms underlying progressive scarring of the liver (fibrogenesis) have been explored and consolidated in the past few years [1, 3]. Since many cell types are involved in liver fibrosis, including HSCs, SECs and KCs, targeting only one cell type may be insufficient [25].

Angiogenesis is a basic change occurring during repair by granulation tissue [26] and is a hypoxia-stimulated, growth factor-dependent process involving the formation of new vascular structures from pre-existing blood vessels [27]. Hepatocellular hypoxia and angiogenesis have been found to accompany fibrogenesis after liver injury, with hypoxia contributing directly to the fibrosis progression [28]. Following CCl4-induced liver injury in mice, anti-angiogenic agents have been found to ameliorate fibrosis and improve survival by promoting parenchymal liver regeneration [29]. However, antiangiogenic therapy, consisting of pharmacological inhibition of integrins αvβ3, was found to promote fibrosis progression, both in experimental biliary (portal) and panlobular hepatic fibrosis [13]. Nevertheless, integrin inhibition had antifibrotic effects on isolated HSCs, which up-regulate this receptor upon activation. Although we found that sorafenib alone significantly inhibited the increases in vWF, CD31, VEGF, Ang1 and VACM1 expression observed in DMN-induced liver fibrosis, sorafenib could not decrease significantly Col1 (α1) expression or Hyp content. This is not consistent with others [30]. Such a difference may be due to the fact that the dose of sorafenib used here is low. On the other hand, only reduction on angiogenesis, one important factor in liver fibrosis, is not sufficient to inhibit fibrosis development [31]. Meanwhile these results indicating that other pathological factor, such as pro-inflammatory and pro-fibrotic also play a key role in liver fibrosis.

Previously we reported that KCs are associated with apoptosis, inflammation and fibrosis [20]. The role of macrophages in the pathogenesis of liver fibrosis has been investigated using specific KC blocking agents such as GdCl3. Surprisingly, although we found that GdCl3 inhibited KC activation and the expression of pro-inflammatory cytokines, it did not improve liver function or liver Hyp content significantly, in contrast to previous findings [14]. Since liver fibrosis arises from the interaction of many pathological factors, inhibiting KC activation alone was not enough to suppress liver fibrosis development; for example, GdCl3 had not significantly effect on the expression of angiogenic-associated factors, such as vWF, CD31, and VCAM. Furthermore, GdCl3 has been found to enhance macrophage activation and the expression of pro-inflammatory cytokines in the lung. Based on these reasons, we could conclude that GdCl3 has very limited effect on liver fibrosis [16].

Liver fibrosis is believed to be reversible through the apoptosis of activated HSCs and the degradation of ECM proteins [23]. Treatment with sorafenib has been found to reduce portal pressure and angiogenesis in DMN- and BDL-treated rats [32]. In addition, sorafenib was found to inhibit the proliferation of various tumor cells and to induce their apoptosis by targeting the tyrosine kinase associated with PDGFR-β [33, 34]. In addition, the induction of apoptosis was found to be accompanied by the down-regulation of cyclins and Cdks in HSCs [35]. In contrast, other studies reported that sorafenib could not improve liver fibrosis in rats [13, 36]. Taken together, these results suggest that sorafenib has limited effects on liver fibrosis.

Understanding of the pathogenesis of human liver fibrosis has progressed significantly over the past 10–15 years [37, 38]. Indeed, the *in vivo* microenvironment is important in regulating HSC activation and function. In this complex environment, KCs and liver SECs modulate inflammation and angiogenesis during the development of liver fibrosis. KCs produce TNF-α, while liver SECs secrete VEGF, activating HSCs. These cells produce ECM proteins, particularly collagen I, thus contributing to hepatic injury. The combination of two fibrosis inhibitors may be superior to each alone [39]. The mechanism of combination treatment in DMN-treated liver fibrosis should be further investigated.

In summary, the data presented in the present study demonstrates that sorafenib significantly inhibited angiogenesis and related factors, and that GdCl3 reduced KC activation and inhibited proinflammatory cytokines. The combination of sorafenib plus GdCl3 may significantly hepatic fibrosis by inhibiting angiogenesis, proinflammatory cytokines, and the interactions of HSCs, SECs and KCs.

## Conclusion

Sorafenib plus GdCl3 can suppress collagen accumulation, suggesting that this combination may be a potential therapeutic strategy in the treatment of liver fibrosis.

## Additional file

Additional file 1: Table S1. Primers used for PCR. **Table S2.** Effects of sorafenib plus GdCl3 on body, liver and spleen weights in DMN-induced rat liver fibrosis (mean ± sd). **Table S3.** the effects of sorafenib, GdCl3, and sorafenib plus GdCl3 on liver function. (DOCX 123 kb)

## Abbreviations

ALB: albumin
ALT: alanine aminotransferase
α-SMA: alpha-smooth muscle actin
AST: aspartate aminotransferase
BSA: bovine serum albumin
DMN: dimethylnitrosamine
GdCl3: gadolinium chloride
HCC: hepatocellular carcinoma
HSC: hepatic stellate cells
Hyp: hydroxyproline
KCs: kupffer cells
MMPs: matrix metalloproteinases
PBS: phosphate-buffered saline
PDGFR: platelet-derived growth factor receptor
ROS: reactive oxygen species
SECs: sinusoidal endothelial cells
VEGFR: vascular endothelial growth factor receptor
